The article "The Basics of Bacteriuria: Strategies of Microbes for Persistence in Urine" was published in 2016. Journal: Front Cell Infect Microbiol.

# The Basics of Bacteriuria: Strategies of Microbes for Persistence in Urine

**DOI:** 10.3389/fcimb.2016.00014

**Published:** 2016-02-08

**Authors:** Deepak S. Ipe, Ella Horton, Glen C. Ulett

**Affiliations:** School of Medical Science, Menzies Health Institute Queensland, Griffith UniversityGold Coast, QLD, Australia

**Keywords:** bacteriuria, asymptomatic bacteriuria, urinary tract infection, urine, urinalysis, uropathogen, synthetic human urine, artificial urine

## Abstract

Bacteriuria, the presence of bacteria in urine, is associated with asymptomatic, as well as symptomatic, urinary tract infection (UTI). Bacteriuria underpins some of the dynamics of microbial colonization of the urinary tract, and probably impacts the progression and persistence of infection in some individuals. Recent molecular discoveries *in vitro* have elucidated how some key bacterial traits can enable organisms to survive and grow in human urine as a means of microbial fitness adaptation for UTI. Several microbial characteristics that confer bacteruric potential have been identified including *de novo* synthesis of guanine, relative resistance to D-serine, and catabolism of malic acid. Microbial characteristics such as these are increasingly being defined through the use of synthetic human urine (SHU) *in vitro* as a model to mimic the *in vivo* environment that bacteria encounter in the bladder. There is considerable variation in the SHU model systems that have been used to study bacteriuria to date, and this influences the utility of these models. In this review, we discuss recent advances in our understanding of bacteruric potential with a focus on the specific mechanisms underlying traits that promote the growth of bacteria in urine. We also review the application of SHU in research studies modeling UTI and discuss the chemical makeup, and benefits and limitations that are encountered in utilizing SHU to study bacterial growth in urine *in vitro*.

## Introduction: bacteriuria and urinary tract infection

“Asymptomatic Bacteriuria” (ABU or ASB) is synonymous with asymptomatic Urinary Tract Infection (UTI) in defining the isolation of a specified semi-quantitative count of bacteria in an appropriately collected urine specimen from a person without signs or symptoms related to UTI (Rubin et al., 1992; Nicolle et al., 2005). Bacteriuria is a marker for symptomatic UTI (sUTI) and assists in grading the severity of infection. Establishment of bacteriuria depends on entry of an organism with bacteruric potential into the urinary tract and can persist for months or years. Bacteruric potential encompasses microbial survival, growth, and re-growth in urine, and endurance of host defense mechanisms including dilution, voiding, frequent flushing (O'grady and Cattell, 1966a,b), and antimicrobial constituents such as Tamm-Horsfall glycoprotein (aka uromodulin), and P blood group antigen (Hand et al., 1971; Lomberg et al., 1983; Bates et al., 2004). Bacteruric potential can thus influence the persistence of ABU and sUTI. Here, we analyze the differences in microbial strategies used for growth in urine and the methods for modeling bacteriuria using synthetic human urine (SHU).

## Microbial bacteruric potential and host dynamics

Recent reviews have focused on the pathogenesis of acute sUTI (Nielubowicz and Mobley, 2010; Hannan et al., 2012; Ulett et al., 2013), and ABU (Ipe et al., 2013; Schneeberger et al., 2014) and will not be revisited here. We will focus on bacteriuria specifically; the progression of which depends on microbe traits as well as host factors. Most individuals who suffer persistent UTI do not harbor the same strain of organism over time (Hooton et al., 2000), implying that turnover of causal organisms is dynamic. Replacement of colonizing strains during bacteriuria has been studied for *Escherichia coli*, the most common cause of ABU (Ipe et al., 2013). Long-term bacteriuria appears to select for attenuated virulence phenotypes of colonizing strains (Salvador et al., 2012). While most microbes are killed by urine, different organisms have distinct bacteruric potential. Several traits can affect microbial growth in urine. Antibiotics stop the progression of bacteriuria (Schneeberger et al., 2012) but patients infected with *E. coli* experience re-colonization with the same or similar organism at high rates (Dalal et al., 2009). This highlights the dynamic nature of bacteriuria and the role of therapeutic intervention [that is not recommended as routine for ABU (Nicolle, 2014)]. Other factors that are associated with the promotion of long-term bacteriuria are defects in immune signaling pathways such as TLRs (Ragnarsdóttir and Svanborg, 2012). Thus, persistence of bacteriuria relates to microbial bacteruric potential and host characteristics/dynamics including genetic immunodeficiency, re-current infection or strain replacement, and antibiotic therapy.

### Microbial metabolism and growth fitness in urine: knowledge from *E. coli*

The progression of bacteriuria depends on a microbes' ability to survive the antimicrobial properties of urine. Urine survival and growth maintains a pool of colonizing organisms regardless of adherence to host cells, and urodynamic properties (urine flow rates, voiding) that differ between individuals (Wullt et al., 1998). Non-voided organisms in residual urine can grow and re-grow to maintain infection. Discoveries using ABU microbes have shaped our understanding of how bacteriuria progresses. ABU *E. coli* strain 83972 displays robust fitness for urine growth (Klemm et al., 2006; Roos et al., 2006b) though this is not a defining feature of all ABU *E. coli*, and is observed in some uropathogenic *E. coli* (UPEC) (Stamey and Mihara, 1980; Alteri and Mobley, 2007; Alteri et al., 2009; Aubron et al., 2012). Poor urine growth has been reported for some fecal *E. coli* isolates (Stamey and Mihara, 1980; Gordon and Riley, 1992). ABU *E. coli* 83972 has been investigated as a prophylactic means to treat acute sUTI (Hull et al., 2000; Wullt, 2003; Roos et al., 2006a; Sundén et al., 2006; Klemm et al., 2007; Watts et al., 2012a). The metabolic basis for urine growth of ABU *E. coli* 83972 involves transport and degradation pathways for galacturonate, glucuronide and galactonate (Roos et al., 2006b), and antioxidant defense mechanisms (Aubron et al., 2012); the details are described elsewhere (Roos et al., 2006a,b). More recently, analysis of ABU *E. coli* 83972 re-isolates indicated marked versatility of metabolic pathways in urine, including utilization of amino acids, hexuronates or (deoxy-) ribonucleosides as an adaptation to individual hosts (Zdziarski et al., 2010). This underlines the metabolic versatility of *E. coli* in urine in response to host-specific metabolic constraints. *guaA* and *argC* were shown to be critical for urine growth and a lack of urinary guanine (or derivatives), combined with an inability of *E. coli* to synthesize these compounds *de novo*, prevents the synthesis of other guanine (or derivative)-dependent products that are required for growth (Russo et al., 1996). Separate from guanine, *argC* and *carAB* mutants had reduced growth in urine in a *E. coli* transposon mutagenesis study, illustrating a role for arginine metabolism (Vejborg et al., 2012).

### Knowledge from bacteria other than *E. coli*

Clinical isolates of *Enterococcus faecalis, Proteus vulgaris, Pseudomonas aeruginosa, Klebsiella pneumoniae, Staphylococcus saprophyticus*, and *Streptococcus agalactiae* have been shown to grow in human urine (Table 1). However, little is known about the mechanisms used by these organisms for urine growth. For *E. faecalis* there are some similarities to *E. coli*; *E. faecalis* expresses multiple virulence genes in urine (Shepard and Gilmore, 2002) including genes for iron transport (Vebø et al., 2010). Iron utilization mechanisms have been reported in urine growth assays with *E. coli* (Watts et al., 2012b). Limiting manganese may be important in restricting *E. faecalis* urine growth (Järvisalo et al., 1992; Low et al., 2003; Vebø et al., 2010). In contrast to activation of pathways described for *E. coli, E. faecalis* activates citrate and aspartate metabolic pathways, and represses glucose uptake (Vebø et al., 2010). Human urine contains more citrate than glucose (Shaykhutdinov et al., 2009; Wishart et al., 2009; Bouatra et al., 2013), which could promote growth of *E. faecalis*. However, human urine is highly variable in chemical constituency and different levels of components such as glucose may influence microbial growth; for example, glucosuria enhances growth of *E. coli*. *E. faecalis* also upregulates genes for utilization of sucrose (and perhaps fructose), another constituent of urine (Tasevska et al., 2005; Bouatra et al., 2013). Other *E. faecalis* genes thought to function in urine growth include those related to import of phosphorylated sugars and glycerol, N-acetyl glucosamine metabolism (Vebø et al., 2010), cysteine synthase, and pathways for conversion of aspartate and α-ketoglutarate to oxaloacetate and glutamate. Urinary aspartate may be used for nitrogen metabolism (Guo and Li, 2009). *E. faecalis* is auxotrophic for multiple amino acids but human urine contains several amino acids including arginine, glutamate, glycine, and leucine (Guo and Li, 2009; Bouatra et al., 2013).

**Table 1:** **Summary of traits that contribute to bacteruric potential in microbes**.

**Trait that confers bacteruric potential**	**Bacterial species**	**References**
Ability to utilize human urine as a substrate for growth	*E. coli*	Gordon and Riley, 1992; Russo et al., 1996; Roesch et al., 2003; Snyder et al., 2004; Johnson et al., 2006; Roos et al., 2006a; Alteri and Mobley, 2007; Klemm et al., 2007; Aubron et al., 2012; Vejborg et al., 2012; Watts et al., 2012b; Hryckowian et al., 2015; King et al., 2015; Shields-Cutler et al., 2015
	*E. faecalis*	Shepard and Gilmore, 2002; Vebø et al., 2010; La Rosa et al., 2012
	*P. vulgaris*	Nickel et al., 1985; Carlsson et al., 2001
	*P. aeruginosa*	Nickel et al., 1985; Carlsson et al., 2001; Storer et al., 2011
	*K. pneumoniae*	Storer et al., 2011; Russo et al., 2015
	*S. saprophyticus*	Sakinç et al., 2009
	*S. agalactiae*	Ipe et al., 2016
Tolerance to high levels of D-serine	*S. saprophyticus*	Sakinç et al., 2009
Requirement for *dsda* for rapid urine growth	*E. coli*	Hryckowian et al., 2015
Capacity for synthesis of guanine-dependent products critical for survival in urine	*E. coli*	Russo et al., 1996
Expression of iron acquisition systems for growth in nutrient limiting environment	*E. coli*	Alteri and Mobley, 2007; Watts et al., 2012b; Shields-Cutler et al., 2015
	*E. faecalis*	Vebø et al., 2010
Osmoadaption, and intracellular accumulation of glycine betaine	*E. coli*	Chambers and Lever, 1996; Deutch et al., 2006
Adaptation of central metabolism to lactate, citrate and amino acids as carbon sources; flux through pyruvate metabolism, TCA cycle	*P. aeruginosa*	Tielen et al., 2013; Berger et al., 2014
Malic acid metabolism	*S. agalactiae*	Ipe et al., 2016

An analysis of metabolic traits of *P. aeruginosa* using synthetic urine revealed adaptation in central metabolism to lactate, citrate, and amino acids as carbon sources, and the induction of amino acid utilization pathways (Tielen et al., 2013). Metabolic flux analysis showed the use of the Entner-Doudoroff pathway with respiratory metabolism, with the pentose phosphate pathway being used exclusively for biosynthesis. Flux through pyruvate metabolism, the tricarboxylic acid cycle, and the glyoxylate shunt was highly variable, and likely caused by adaptive processes in individual strains during infection (Berger et al., 2014).

Phenotype metabolic arrays were recently reported for ABU *S. agalactiae* (Ipe et al., 2016). Comparison with *S. agalactiae* strains that were unable to grow in urine showed that malic acid catabolism was important for growth in urine. Malic acid utilization is related to the malic enzyme metabolic pathway that catalyzes the oxidative decarboxylation of malate (a component of human urine depending on diet) to pyruvate and CO_2_. This is related to malolactic fermentation, a bacterial metabolic process typically associated with wine deacidification (Landete et al., 2010).

### Three ways to survive in urine: resistance, acquisition, and osmoadaption

Urine is naturally antimicrobial; hypertonicity with low pH (averaging ~6.0) and high concentrations of urea inhibit most bacteria (Chambers and Lever, 1996; Kucheria et al., 2005). Nitrite in mildly acidified urine inhibits the growth of some uropathogens (Carlsson et al., 2001), and other abundant proteins such as Tamm-Horsfall glycoprotein are antimicrobial (Raffi et al., 2005; Säemann et al., 2005). Recently, the antimicrobial properties of urine were shown to include specific inhibition of both expression and function of UPEC type 1 pili (Greene et al., 2015), and downregulation of capsule genes (King et al., 2015). Individualistic urinary chemical features can also affect the antimicrobial properties of some antimicrobial urinary proteins such as siderocalin (Shields-Cutler et al., 2015). Bacteria that can endure urine antimicrobial properties do so through various means; for example, *S. saprophyticus* tolerates high concentrations of D-serine, which is abundant in urine and bacteriostatic toward organisms that lack a D-serine deaminase (Cosloy and McFall, 1973; Hryckowian et al., 2015). Iron limitation and the presence iron chelators such as lactoferrin (Weinberg, 1978) compounds the problem of nutritional immunity for microbes (Hood and Skaar, 2012) especially during states of increased iron chelator production (Gonzalez-Chavez et al., 2009; Soler-García et al., 2009). Siderophores confer bacteruric potential to *E. coli* (Håversen et al., 2000; Snyder et al., 2004; Alteri and Mobley, 2007; Hagan and Mobley, 2009; Garcia et al., 2011; Watts et al., 2012b) and several genes encoding factors involved in iron transport are upregulated in *E. faecalis* during urine growth (Vebø et al., 2010). Siderophores may also act as ligands for cations other than iron, such as copper (Chaturvedi et al., 2012). Variable resistance to urinary defense molecules (e.g., nitrite, ascorbic acid) could influence bacteruric potential but little is known beyond the effects of these toward the chemical properties of urine (Carlsson et al., 2001). Finally, many organisms are probably unable to survive the oxygen concentrations encountered in the bladder (Leonhardt and Landes, 1963; Clarke et al., 1985).

Urea is abundant in urine and is antibacterial (Sobel, 1985). Osmoadaptive systems enable some bacteria to survive the stressful hypertonic conditions of urine. Bacterial accumulation of osmotically compatible solutes that are present in urine (e.g., betaines) confers bacteruric potential by effectively enabling microbes to resist dehydration (Chambers and Lever, 1996; Deutch et al., 2006). Osmoadaptive systems respond to changes in tonicity in urine, and support survival by counteracting low pH, high urea concentrations and hypertonicity (Chambers and Lever, 1996). For *E. coli*, glycine betaine is a central osmoprotectant to resist urea toxicity, and its accumulation is essential to adaptive responses to osmotic stress (Kunin et al., 1992; Chambers and Lever, 1996). *E. coli* increases the activity of potassium transport systems that encompass TrkG, TrkH, and Kup (Meury et al., 1985), or Kdp (Laimins et al., 1978) to counteract osmotic stress. Other systems involve trehalose as an organic osmolyte; its induction is triggered in conditions of high potassium (and glutamate) (Strøm and Kaasen, 1993), and its accumulation elicits the release of potassium from the cell (Dinnbier et al., 1988). This might aid growth since trehalose can be used as a carbon source (Gutierrez et al., 1989; Styrvold and Strøm, 1991). OmpR regulates osmoadaptive genes in *E. coli* (Barron et al., 1986). Osmotic stress suppresses the expression of fimbriae and flagellin (Kunin et al., 1994, 1995). Future studies of bacteria other than *E. coli* that can grow in urine will elucidate additional mechanisms of resistance to urinary antimicrobial properties, nutrient acquisition and metabolism, and osmoadaption.

### Between a rock and a hard-place: the bladder mucosa-lumen interface of immune surveillance and bacteriuria

Inflammation is a critical part of sUTI pathogenesis (Hannan et al., 2012; Ulett et al., 2013) and involves thousands of genes that drive antibacterial responses within hours of infection (Duell et al., 2012; Tan et al., 2012; Carey et al., 2016). For example, antimicrobial peptides produced by the bladder are important for protection against infection (Chromek et al., 2006). Microbes must survive these inflammatory events. Urine is a “Hard-place” for microbes to survive, as discussed above. Tissue inflammation in the bladder represents a “rock” of antimicrobial responses for defense against UTI and, for ABU, can encompass pyuria, cytokine release (IL-1α, -6, and -8), and antibody production, which has been documented in elderly adults, as reviewed elsewhere (Nicolle, 1997). Excessive inflammation may contribute to chronic sUTI (Hannan et al., 2010) and some acute sUTI symptoms have been linked to specific inflammatory events (Rudick et al., 2010). However, the benign, minimally inflammatory nature of ABU is reflected in the lack of morbidity in individuals who do not receive therapy (Nicolle, 1997, 1999; Ariathianto, 2011). Details of how ABU bacteria induce and minimize inflammation offer insight into how microbial modulation of host defense may promote bacteriuria. ABU *E. coli* minimizes inflammation by averting adherence due to a lack of fimbriae expression; this limits immune activation (Roos et al., 2006b) and results in long-term ABU (Arthur et al., 1989; Andersson et al., 1991). Grönberg-Hernandez et al. showed that ABU *E. coli* activates IRF3 and TLR4-dependent signaling, however, triggering a response that depends on host genetic background (Grönberg-Hernández et al., 2011); the IRF3-dependent signaling pathway is critical for distinguishing pathogens from the normal flora (Fischer et al., 2010). TLR4 senses P-fimbriated *E. coli* (Frendéus et al., 2001), and TLR4 mutations may favor ABU by impeding innate responses (Svanborg et al., 2006). This raises the question of whether ABU may influence subsequent encounter(s) with other uropathogens. One study on streptococcal UTI showed an influence on the severity of subsequent *E. coli* UTI in mice (Kline et al., 2012). Thus, immune activation triggered by ABU might affect subsequent sUTI caused by diverse pathogens. These data offer some parallel to clinical observations that patients with *E. coli* ABU suffer re-colonization at high rates following therapy (Dalal et al., 2009).

## Modeling bacteriuria *in vitro*: synthetic human urine (SHU)

Urine is unique from a microbial perspective and its chemical makeup, distinct from all other bodily fluids, has been modeled for studying the growth of microbes for 50 years (O'grady and Pennington, 1966). Urine has a low pH and a high osmolality due to the presence of salts and urea (Kucheria et al., 2005; Sheewin, 2011). The peptides, proteins, and organic acids present in urine may be metabolized by microbes (Decramer et al., 2008). Urine is dynamic in flow rate and composition, which changes subject to diet, age, gender and health status, and disease. Decreased levels of THP, for example, are associated with diabetes (Torffvit and Agardh, 1993) and infection (Ronald and Ludwig, 2001). Data on microbial traits that afford bacteruric potential have, in many cases, been derived from studies using SHU. Eight original SHU media recipes were described between 1971 and 2010: as summarized according to research application and composition in Table 2.

**Table 2:** **Original and subsequent studies using Synthetic Human Urine (SHU) (A), and related SHU constituents, and proposed composite SHU (B)**.

**A. Original study^1^**	**Focus of the research application**	**Microbes or cell types**	**Relevance**	**Reference(s) citing the original study**
1. Physiology (Aurora et al., 1980)	Understanding the development of calcium oxalate monohydrate precipitation	N/A	Urolithiasis	Mayrovitz and Sims, 2001
2. Infection (Brooks and Keevil, 1997)	Development of SHU to investigate the growth of urinary pathogens	*E. coli, P. aeruginosa, P. mirabilis, S. epidermidis, C. albicans*	UTI	Darouiche et al., 2008; Wernli et al., 2013; Azevedo et al., 2014; Lehman and Donlan, 2015; Wilks et al., 2015
3. Physiology (Burns and Finlayson, 1980)	Description of standard SHU for *in vitro* urolithiasis assays	N/A	Urolithiasis	Brown et al., 1989; Rodgers and Wandt, 1991; Opalko et al., 1997; Mayrovitz and Sims, 2001; Christmas et al., 2002; ^2^(Isaacson, 1969; Barker et al., 1974; Rose, 1975; Miller et al., 1977; Doremus et al., 1978; Gardner and Doremus, 1978)
4. Cell Biology (Chutipongtanate and Thongboonkerd, 2010)	Comparison of multiple SHU media, and study in epithelial cell culture assays	Kidney epithelial cells	Cell Biology	^2^^,^^3^(Brown et al., 1989; Brooks and Keevil, 1997; Opalko et al., 1997; Grases and Llobera, 1998; Mayrovitz and Sims, 2001; Christmas et al., 2002); (Samaranayake et al., 2014)
5. Infection and Physiology (Griffith et al., 1976)	Investigation of infection-induced urinary stones	*E. coli, P. aeruginosa, P. mirabilis, Citrobacter koseri, Proteus rettgeri, Providencia stuartii, Morganella morganii, Klebsiella oxytoca*,	UTI, and Urolithiasis	Davis et al., 1989, 1991; Martino et al., 2003; Dalhoff et al., 2011; Phuengkham and Nasongkla, 2015. ^4^Cited by: (Domergue et al., 2005; Mabbett et al., 2009; Ong et al., 2009, 2010). ^4^Cited by: (Watts et al., 2010; Jain et al., 2007). ^4^Cited by: (Silva et al., 2010; Rane et al., 2014; Negri et al., 2015); ^2^(Robertson et al., 1968)
6. Infection (Minuth et al., 1976)	Measurement of the antimicrobial efficacy of gentamicin in SHU	*E. coli, P. aeruginosa*	UTI	Mansouri and Darouiche, 2008; Sako et al., 2014
7. Physiology (Putnam et al., 1971)	Characterization of urinary constituents	N/A	General	No citations published
8. Physiology (Gardner and Doremus, 1978)	Study of calcium oxalate crystallization	N/A	Urolithiasis	Robertson et al., 1981. ^4^Cited by: (Robertson and Scurr, 1986)
**B. Constituent**	**(n)**^5^	**Mean Conc. (Range)**^6^	**Composite**^7^	**References Citing Constituent**
NaCl	8/8	113.3 (54–231) mM	100 mM	Griffith et al., 1976; Minuth et al., 1976; Gardner and Doremus, 1978; Aurora et al., 1980; Burns and Finlayson, 1980; Robertson and Scurr, 1986; Brooks and Keevil, 1997; Chutipongtanate and Thongboonkerd, 2010
Na_2_SO_4_	8/8	17.0 (9.0–155,800) mM	17.0 mM	Griffith et al., 1976; Minuth et al., 1976; Gardner and Doremus, 1978; Aurora et al., 1980; Burns and Finlayson, 1980; Robertson and Scurr, 1986; Brooks and Keevil, 1997; Chutipongtanate and Thongboonkerd, 2010
pH	7/8	6.0 (5.7–7.2)	5.5–6.0	Griffith et al., 1976; Minuth et al., 1976; Gardner and Doremus, 1978; Burns and Finlayson, 1980; Robertson and Scurr, 1986; Brooks and Keevil, 1997; Chutipongtanate and Thongboonkerd, 2010
Urea	6/8	281 (170–500) mM	280 mM	Griffith et al., 1976; Minuth et al., 1976; Gardner and Doremus, 1978; Aurora et al., 1980; Brooks and Keevil, 1997; Chutipongtanate and Thongboonkerd, 2010
KCl	6/8	58.5 (21.5–162.7) mM	38.0 mM	Griffith et al., 1976; Minuth et al., 1976; Aurora et al., 1980; Burns and Finlayson, 1980; Robertson and Scurr, 1986; Chutipongtanate and Thongboonkerd, 2010
CaCl_2_	6/8	5.3 (2.5–12.0) mM	4.0 mM	Griffith et al., 1976; Minuth et al., 1976; Burns and Finlayson, 1980; Robertson and Scurr, 1986; Brooks and Keevil, 1997; Chutipongtanate and Thongboonkerd, 2010
Creatinine	5/8	8.7 (4.0–13.2) mM	9.0 mM	Griffith et al., 1976; Minuth et al., 1976; Aurora et al., 1980; Brooks and Keevil, 1997; Chutipongtanate and Thongboonkerd, 2010
Na_3_C_6_H_5_O_7_	5/8	3.4 (2.2–5.0) mM	3.4 mM	Griffith et al., 1976; Minuth et al., 1976; Burns and Finlayson, 1980; Robertson and Scurr, 1986; Chutipongtanate and Thongboonkerd, 2010
NH_4_Cl	5/8	36.6 (15.0–86.8) mM	20.0 mM	Griffith et al., 1976; Minuth et al., 1976; Robertson and Scurr, 1986; Brooks and Keevil, 1997; Chutipongtanate and Thongboonkerd, 2010
MgSO_4_	5/8	3.2 (2.0–5.9) mM	3.2 mM	Aurora et al., 1980; Burns and Finlayson, 1980; Robertson and Scurr, 1986; Brooks and Keevil, 1997; Chutipongtanate and Thongboonkerd, 2010
Na_2_C_2_O_4_	5/8	0.38 (0.1–1.2) mM	0.18 mM	Griffith et al., 1976; Minuth et al., 1976; Burns and Finlayson, 1980; Chutipongtanate and Thongboonkerd, 2010
NaH_2_PO_4_	4/8	20.9 (3.6–43.6) mM	3.6 mM	Aurora et al., 1980; Burns and Finlayson, 1980; Robertson and Scurr, 1986; Chutipongtanate and Thongboonkerd, 2010
Na_2_HPO_4_	4/8	6.5 (6.1–186,800) mM	6.5 mM	Gardner and Doremus, 1978; Aurora et al., 1980; Robertson and Scurr, 1986; Chutipongtanate and Thongboonkerd, 2010
KH_2_PO_4_	3/8	16.0 (7.0–20.6) mM	16.0 mM	Griffith et al., 1976; Minuth et al., 1976; Brooks and Keevil, 1997
C_5_H_4_N_4_O_3_	3/8	0.6 (0.4–1.0) mM	0.6 mM	Aurora et al., 1980; Brooks and Keevil, 1997; Chutipongtanate and Thongboonkerd, 2010
NaHCO_3_	2/8	13.5 (2.0–25.0) mM	13.5 mM	Brooks and Keevil, 1997; Chutipongtanate and Thongboonkerd, 2010
MgCl_2_.6H_2_O	2/8	3.2 (3.2) mM	3.2 mM	Griffith et al., 1976; Minuth et al., 1976
Osmolality	2/8	586 (446–725) mOsm/kg	600 mOsm/kg	Minuth et al., 1976; Chutipongtanate and Thongboonkerd, 2010
C_6_H_8_O_7_	2/8	1.7 (1.4–2.0) mM	–	Aurora et al., 1980; Brooks and Keevil, 1997
TSB^8^	2/8	2.0% (1.0–5.0%) (v/v)	–	Griffith et al., 1976; Minuth et al., 1976; Torzewska et al., 2003, 2014; Torzewska and Rózalski, 2014, 2015
NH_3_OH	1/8	17.1 mM	–	Aurora et al., 1980
C_9_H_9_NO_3_	1/8	2.8 mM	–	Aurora et al., 1980
K_2_HPO_4_	1/8	7.0 mM	–	Brooks and Keevil, 1997
C_3_H_6_O_3_	1/8	1.1 mM	1.1 mM	Brooks and Keevil, 1997
FeSO_4_.7H_2_O	1/8	0.005 mM	0.005 mM	Brooks and Keevil, 1997
K_3_C_6_H_5_O_7_	1/8	2752000 mM	–	Gardner and Doremus, 1978
Mg(NO_3_)_2_	1/8	2.5 mM	–	Gardner and Doremus, 1978
Peptone^8^	1/8	0.1% (w/v)	–	Brooks and Keevil, 1997
Yeast extract^8^	1/8	0.0005% (w/v)	–	Brooks and Keevil, 1997
Glucose	0/8	1.0% (0.3–2.0%) (w/v)	–	Uppuluri et al., 2009; Silva et al., 2010; Negri et al., 2012, 2015
Sucrose	0/8	0.002% (w/v)	–	Wernli et al., 2013
Lactose	0/8	0.002% (w/v)	–	Wernli et al., 2013
LB^8^	0/8	3.5% (2.5–5.0%) (v/v)	–	Martino et al., 2003; Domergue et al., 2005; Wenzler-Röttele et al., 2006; Ong et al., 2009, 2010; Ipe et al., 2016
Dextrose^8^	0/8	3.4% (0.3–8.0%) (w/v)	–	Domergue et al., 2005; Jain et al., 2007; Negri et al., 2011
THB^8^	0/8	2.5% (v/v)	–	Ipe et al., 2016
YNB^8^	0/8	5.0% (5.0–5.0%) (v/v)	–	Jain et al., 2007; Uppuluri et al., 2009
SC Broth^8^	0/8	5.0% (v/v)	–	Domergue et al., 2005
Nutrient Broth^8^	0/8	1.2% (0.4–2.0%) (v/v)	–	Wenzler-Röttele et al., 2006; Sako et al., 2014
Gelatine^8^	0/8	1.0% (w/v)	–	Wenzler-Röttele et al., 2006
Casamino Acids, Bacto^8^	0/8	–	0.1% (v/v)	

1 Original study of Robinson et al. (1984) cited by Lee et al. (1995) does not provide a recipe;

2 Reference(s) included in original study (minimal recipe details in reference citing original study);

3 Original studies of Brooks and Keevil (1997) and Grases and Llobera (1998) cited by Chutipongtanate and Thongboonkerd (2010) provide a recipe;

4 Cited by: these references cite the immediate preceding reference rather than the original study;

5 The number of original studies (n/8) that defined the component in their SHU recipe;

6 Refers to Average Concentration, and (Concentration Range). Study of Robertson and Scurr (1986) was used to calculate Mean Concentration, and (Concentration Range) instead of Original Study of Putnam et al. (1971) because Putnam et al. (1971) does not provide a SHU recipe;

7 Proposed Composite SHU Media Concentrations are based on average values in referenced studies, and most compare closely to the typical human urine chemical composition as reported in Putnam et al. (1971) (e.g., NaCl 137 mM, Urea 223 mM, KCl 22 mM, Creatinine 13.3 mM, MgSO_4_ 6.5 mM). In some cases (e.g., Na_2_HPO_4_, Na_2_SO_4_, KCl, Na_2_C_2_O_4_) the means and composite SHU values are chosen to exclude extreme upper range values from Gardner and Doremus (1978), Robertson and Scurr (1986).

8 References cited for components are original studies only, excepting for these components, for which all published studies using these components are cited. The proposed composite SHU omits Trypticase Soy Broth (TSB), peptone, LB, THB, and Nutrient Broth (undefined), Yeast Nitrogen Base (YNB) and Synthetic Complete (SC) Broth (for fungi), but includes 0.1% v/v Casamino Acids, Bacto (20% stock solution; BD) to attain a chemically defined minimal SHU medium, with the addition of 0.2% v/v (10% stock solution) yeast extract as a proposed supplement for fastidious bacteria including Streptococcus, or 2.0% w/v dextrose and 5.0% v/v YNB for fungi.

SHU offers several advantages compared to normal human urine collected from healthy adults for research assays *ex vivo*; it avoids the issue of variable chemical composition encountered with fresh human urine; variation in urinary constituents between individuals (Bouatra et al., 2013) is a challenge for standardizing research studies. Methods for “normalizing” fresh human urine include pooling samples and adjusting dilution/concentration according to creatinine concentration, specific gravity, and osmolality. The most widely used method is creatinine adjustment (Barr et al., 2005), however no bacteriuria research studies to date have applied these methods for normalizing, and the effects on data interpretation are unknown. Volume limits have been difficult for some studies (Davis et al., 1982). As a surrogate model, the benefits of SHU are defined by how closely it can reflect the chemical complexity of fresh human urine. Urine from a healthy adult contains glucose (0.2–0.6 mM) (Shaykhutdinov et al., 2009), creatine (0.38–55.6 mM; Barr et al., 2005; Shaykhutdinov et al., 2009), and glycine with low levels of other amino acids such as D-serine (Huang et al., 1998; Pätzold et al., 2005), histidine, glutamine, methionine, proline, glutamate, arginine, cysteine, and branched chain amino acids (Guo and Li, 2009; Vebø et al., 2010). It contains trace fatty acids, citrate (1.0–2.0 mM) (Wishart et al., 2009), sucrose (70–200 μM) (Tasevska et al., 2005), and manganese (nM range) (Järvisalo et al., 1992).

To standardize SHU composition for bacteriuria studies, we propose a composite SHU medium recipe (Table 2), and compare this to descriptions of “typical human urine” (Putnam et al., 1971; Bouatra et al., 2013). Examples of supplements to previously used SHU formulations include Lysogeny Broth (LB), Todd-Hewitt Broth (THB), and dextrose for fungi such as *Candida* sp. (Table 2). The proposed composite SHU medium omits chemically undefined components such as LB to provide chemical definition, is easily prepared, inexpensive, and chemically stable. However, it is also not without its limitations; it excludes some natural constituents of human urine such as hormones, iron chelators, and pyrophosphates that could influence microbial growth. The relative concentrations of some urinary constituents differ between males and females (e.g., less calcium and oxalate, more citrate excretion in women, more creatinine in men; Ryall et al., 1987; Sarada and Satyanarayana, 1991; Bouatra et al., 2013) and the proposed composite SHU does not account for these differences. Nonetheless, as a balance between feasibility, logistics, and economy the proposed composite SHU medium should be of value to standardize future bacteriuria studies; importantly, studies will now need to validate the proposed composite SHU medium using a range of relevant bacteria, and in particular, analyze the need for supplements (e.g., yeast extract) to support the growth of fastidious organisms such as streptococci.

## Conclusions and future directions

A capacity of microorganisms for urine growth may aid in establishing long-term bacteriuria and is relevant to many microbial species. New discoveries on immune activation by ABU show this form of infection does not exist entirely under the radar of immune surveillance. Continued use of SHU for *in vitro* studies will drive new discoveries on how bacteriuria progresses and how this may influence subsequent infection. Future work needs to address multiple areas; including (1) validation of the proposed composite SHU medium using a range of relevant bacteria; (2) defining differences in “significant” bacteriuria for different organisms and the implications of bacteruric potential toward such definitions; (3) lifestyle adaptations, other than those described for D-serine, guanine, malic acid, and iron acquisition that aid microbial bacteruric potential; (4) the molecular basis of urine growth in non-*E. coli* organisms; how ABU interfaces with host immune mechanisms for different organisms (and among distinct patient populations); (5) differences in male vs. female urine composition, in particular hormones (and whether this influences bacterial growth); and (6) how ABU impacts on subsequent UTI including comparisons of immune responses to ABU caused by organisms other than *E. coli*. How effective ABU might be as a prophylactic approach against sUTI continues to be a topic for future investigation. More importantly, studies aimed at defining bacterial mechanisms that are critical for growth in urine are essential in the context of providing a foundation for novel treatment and preventive strategies.

## Author contributions

DI, EH, and GU conceived of the study, analyzed the literature, and wrote the manuscript.

### Conflict of interest statement

The authors declare that the research was conducted in the absence of any commercial or financial relationships that could be construed as a potential conflict of interest.

## References

[B1] AlteriC. J.MobleyH. L. (2007). Quantitative profile of the uropathogenic *Escherichia coli* outer membrane proteome during growth in human urine. Infect. Immun. 75, 2679–2688. 10.1128/IAI.00076-0617513849PMC1932884

[B2] AlteriC. J.SmithS. N.MobleyH. L. (2009). Fitness of *Escherichia coli* during urinary tract infection requires gluconeogenesis and the TCA cycle. PLoS Pathog. 5:e1000448. 10.1371/journal.ppat.100044819478872PMC2680622

[B3] AnderssonP.EngbergI.Lidin-JansonG.LincolnK.HullR.HullS. (1991). Persistence of *Escherichia coli* bacteriuria is not determined by bacterial adherence. Infect. Immun. 59, 2915–2921.187991710.1128/iai.59.9.2915-2921.1991PMC258113

[B4] AriathiantoY. (2011). Asymptomatic bacteriuria - prevalence in the elderly population. Aust. Fam. Physician 40, 805–809. 22003486

[B5] ArthurM.JohnsonC. E.RubinR. H.ArbeitR. D.CampanelliC.KimC.. (1989). Molecular epidemiology of adhesin and hemolysin virulence factors among uropathogenic *Escherichia coli*. Infect. Immun. 57, 303–313. 256325410.1128/iai.57.2.303-313.1989PMC313098

[B6] AubronC.GlodtJ.MatarC.HuetO.BorderieD.DobrindtU.. (2012). Variation in endogenous oxidative stress in *Escherichia coli* natural isolates during growth in urine. BMC Microbiol. 12:120. 10.1186/1471-2180-12-12022727065PMC3479029

[B7] AuroraA. L.RaoA. S.SrimathiV. (1980). Effects of constituents of artificial urine on spontaneous precipitation of calcium oxalate monohydrate (whewellite). Ind. J. Med. Res. 72, 273–283. 7228164

[B8] AzevedoA. S.AlmeidaC.MeloL. F.AzevedoN. F. (2014). Interaction between atypical microorganisms and *E. coli* in catheter-associated urinary tract biofilms. Biofouling 30, 893–902. 10.1080/08927014.2014.94417325184430

[B9] BarkerL. M.PallanteS. L.EisenbergH.JouleJ. A.BeckerG. L.HowardJ. E. (1974). Simple synthetic and natural urines have equivalent anticalcifying properties. Invest. Urol. 12, 79–81. 4835493

[B10] BarrD. B.WilderL. C.CaudillS. P.GonzalezA. J.NeedhamL. L.PirkleJ. L. (2005). Urinary creatinine concentrations in the U.S. population: implications for urinary biologic monitoring measurements. Environ. Health Perspect. 113, 192–200. 10.1289/ehp.733715687057PMC1277864

[B11] BarronA.MayG.BremerE.VillarejoM. (1986). Regulation of envelope protein composition during adaptation to osmotic stress in *Escherichia coli*. J. Bacteriol. 167, 433–438. 301586910.1128/jb.167.2.433-438.1986PMC212906

[B12] BatesJ. M.RaffiH. M.PrasadanK.MascarenhasR.LaszikZ.MaedaN.. (2004). Tamm-Horsfall protein knockout mice are more prone to urinary tract infection: rapid communication. Kidney Int. 65, 791–797. 10.1111/j.1523-1755.2004.00452.x14871399

[B13] BergerA.DohntK.TielenP.JahnD.BeckerJ.WittmannC. (2014). Robustness and plasticity of metabolic pathway flux among uropathogenic isolates of *Pseudomonas aeruginosa*. PLoS ONE 9:e88368. 10.1371/journal.pone.008836824709961PMC3977821

[B14] BouatraS.AziatF.MandalR.GuoA. C.WilsonM. R.KnoxC.. (2013). The human urine metabolome. PLoS ONE 8:e73076. 10.1371/journal.pone.007307624023812PMC3762851

[B15] BrooksT.KeevilC. W. (1997). A simple artificial urine for the growth of urinary pathogens. Lett. Appl. Microbiol. 24, 203–206. 10.1046/j.1472-765X.1997.00378.x9080700

[B16] BrownP.AckermannD.FinlaysonB. (1989). Calcium-Oxalate Dihydrate (Weddellite) Precipitation. J. Cryst. Growth 98, 285–292. 10.1016/0022-0248(89)90143-7

[B17] BurnsJ. R.FinlaysonB. (1980). A proposal for a standard reference artificial urine in *in vitro* urolithiasis experiments. Invest. Urol. 18, 167–169. 7410032

[B18] CareyA. J.SullivanM. J.DuellB. L.CrossmanD. K.ChattopadhyayD.BrooksA. J.. (2016). Uropathogenic *Escherichia coli* engages CD14-dependent signaling to enable bladder-macrophage-dependent control of acute urinary tract infection. J. Infect. Dis. 213, 659–668. 10.1093/infdis/jiv42426324782

[B19] CarlssonS.WiklundN. P.EngstrandL.WeitzbergE.LundbergJ. O. (2001). Effects of pH, nitrite, and ascorbic acid on nonenzymatic nitric oxide generation and bacterial growth in urine. Nitric Oxide 5, 580–586. 10.1006/niox.2001.037111730365

[B20] ChambersS. T.LeverM. (1996). Betaines and urinary tract infections. Nephron 74, 1–10. 10.1159/0001892748883013

[B21] ChaturvediK. S.HungC. S.CrowleyJ. R.StapletonA. E.HendersonJ. P. (2012). The siderophore yersiniabactin binds copper to protect pathogens during infection. Nat. Chem. Biol. 8, 731–736. 10.1038/nchembio.102022772152PMC3600419

[B22] ChristmasK. G.GowerL. B.KhanS. R.El-ShallH. (2002). Aggregation and dispersion characteristics of calcium oxalate monohydrate: effect of urinary species. J. Colloid Interface Sci. 256, 168–174. 10.1006/jcis.2002.828312505509

[B23] ChromekM.SlamováZ.BergmanP.KovácsL.PodrackáL.EhrénI.. (2006). The antimicrobial peptide cathelicidin protects the urinary tract against invasive bacterial infection. Nat. Med. 12, 636–641. 10.1038/nm140737001006

[B24] ChutipongtanateS.ThongboonkerdV. (2010). Systematic comparisons of artificial urine formulas for *in vitro* cellular study. Anal. Biochem. 402, 110–112. 10.1016/j.ab.2010.03.03120347669

[B25] ClarkeM.PeadL.MaskellR. (1985). Urinary infection in adult men: a laboratory perspective. Br. J. Urol. 57, 222–226. 10.1111/j.1464-410X.1985.tb06429.x3986460

[B26] CosloyS. D.McFallE. (1973). Metabolism of D-serine in *Escherichia coli* K-12: mechanism of growth inhibition. J. Bacteriol. 114, 685–694. 457469710.1128/jb.114.2.685-694.1973PMC251827

[B27] DalalS.NicolleL.MarrsC. F.ZhangL.HardingG.FoxmanB. (2009). Long-term *Escherichia coli* asymptomatic bacteriuria among women with diabetes mellitus. Clin. Infect. Dis. 49, 491–497. 10.1086/60088319583518PMC2833278

[B28] DalhoffA.StubbingsW.SchubertS. (2011). Comparative *in vitro* activities of the novel antibacterial finafloxacin against selected Gram-positive and Gram-negative bacteria tested in Mueller-Hinton broth and synthetic urine. Antimicrob. Agents Chemother. 55, 1814–1818. 10.1128/AAC.00886-1021245444PMC3067158

[B29] DarouicheR. O.MansouriM. D.GawandeP. V.MadhyasthaS. (2008). Efficacy of combination of chlorhexidine and protamine sulphate against device-associated pathogens. J. Antimicrob. Chemother. 61, 651–657. 10.1093/jac/dkn00618258612

[B30] DavisC. P.ArnettD.WarrenM. M. (1982). Iontophoretic killing of *Escherichia coli* in static fluid and in a model catheter system. J. Clin. Microbiol. 15, 891–894. 704755710.1128/jcm.15.5.891-894.1982PMC272209

[B31] DavisC. P.WagleN.AndersonM. D.WarrenM. M. (1991). Bacterial and fungal killing by iontophoresis with long-lived electrodes. Antimicrob. Agents Chemother. 35, 2131–2134. 10.1128/AAC.35.10.21311759837PMC245340

[B32] DavisC. P.WeinbergS.AndersonM. D.RaoG. M.WarrenM. M. (1989). Effects of microamperage, medium, and bacterial concentration on iontophoretic killing of bacteria in fluid. Antimicrob. Agents Chemother. 33, 442–447. 10.1128/AAC.33.4.4422658791PMC172457

[B33] DecramerS.Gonzalez de PeredoA.BreuilB.MischakH.MonsarratB.BascandsJ. L.. (2008). Urine in clinical proteomics. Mol. Cell. Proteomics 7, 1850–1862. 10.1074/mcp.R800001-MCP20018667409

[B34] DeutchC. E.ArballoM. E.CooksL. N.GomesJ. M.WilliamsT. M.Aboul-FadlT.. (2006). Susceptibility of *Escherichia coli* to L-selenaproline and other L-proline analogues in laboratory culture media and normal human urine. Lett. Appl. Microbiol. 43, 392–398. 10.1111/j.1472-765X.2006.01979.x16965369

[B35] DinnbierU.LimpinselE.SchmidR.BakkerE. P. (1988). Transient accumulation of potassium glutamate and its replacement by trehalose during adaptation of growing cells of *Escherichia coli* K-12 to elevated sodium chloride concentrations. Arch. Microbiol. 150, 348–357. 10.1007/BF004083063060036

[B36] DomergueR.CastañoI.De Las PeñasA.ZupancicM.LockatellV.HebelJ. R.. (2005). Nicotinic acid limitation regulates silencing of Candida adhesins during UTI. Science 308, 866–870. 10.1126/science.110864015774723

[B37] DoremusR. H.TeichS.SilvisP. X. (1978). Crystallization of calcium oxalate from synthetic urine. Invest. Urol. 15, 469–472. 649296

[B38] DuellB. L.CareyA. J.TanC. K.CuiX.WebbR. I.TotsikaM.. (2012). Innate transcriptional networks activated in bladder in response to uropathogenic *Escherichia coli* drive diverse biological pathways and rapid synthesis of IL-10 for defense against bacterial urinary tract infection. J. Immunol. 188, 781–792. 10.4049/jimmunol.110123122184725

[B39] FischerH.LutayN.RagnarsdóttirB.YadavM.JönssonK.UrbanoA.. (2010). Pathogen specific, IRF3-dependent signaling and innate resistance to human kidney infection. PLoS Pathog. 6:e1001109. 10.1371/journal.ppat.100110920886096PMC2944801

[B40] FrendéusB.WachtlerC.HedlundM.FischerH.SamuelssonP.SvenssonM.. (2001). *Escherichia coli* P fimbriae utilize the Toll-like receptor 4 pathway for cell activation. Mol. Microbiol. 40, 37–51. 10.1046/j.1365-2958.2001.02361.x11298274

[B41] GarciaE. C.BrumbaughA. R.MobleyH. L. (2011). Redundancy and specificity of *Escherichia coli* iron acquisition systems during urinary tract infection. Infect. Immun. 79, 1225–1235. 10.1128/IAI.01222-1021220482PMC3067483

[B42] GardnerG. L.DoremusR. H. (1978). Crystal growth inhibitors in human urine. Effect on calcium oxalate kinetics. Invest. Urol. 15, 478–485. 649298

[B43] Gonzalez-ChavezS. A.Arevalo-GallegosS.Rascon-CruzQ. (2009). Lactoferrin: structure, function and applications. Int. J. Antimicrob. Agents 33, 301, e301–e308. 10.1016/j.ijantimicag.2008.07.02018842395

[B44] GordonD. M.RileyM. A. (1992). A theoretical and experimental analysis of bacterial growth in the bladder. Mol. Microbiol. 6, 555–562. 10.1111/j.1365-2958.1992.tb01500.x1560784

[B45] GrasesF.LloberaA. (1998). Experimental model to study sedimentary kidney stones. Micron 29, 105–111. 10.1016/S0968-4328(98)00006-79684348

[B46] GreeneS. E.HibbingM. E.JanetkaJ.ChenS. L.HultgrenS. J. (2015). Human urine decreases function and expression of Type 1 pili in uropathogenic *Escherichia coli*. MBio 6:e00820. 10.1128/mBio.00820-1526126855PMC4488945

[B47] GriffithD. P.MusherD. M.ItinC. (1976). Urease. The primary cause of infection-induced urinary stones. Invest. Urol. 13, 346–350. 815197

[B48] Grönberg-HernándezJ.SundénF.ConnollyJ.SvanborgC.WulltB. (2011). Genetic control of the variable innate immune response to asymptomatic bacteriuria. PLoS ONE 6:e28289. 10.1371/journal.pone.002828922140570PMC3225390

[B49] GuoK.LiL. (2009). Differential 12C-/13C-isotope dansylation labeling and fast liquid chromatography/mass spectrometry for absolute and relative quantification of the metabolome. Anal. Chem. 81, 3919–3932. 10.1021/ac900166a19309105

[B50] GutierrezC.ArdourelM.BremerE.MiddendorfA.BoosW.EhmannU. (1989). Analysis and DNA sequence of the osmoregulated treA gene encoding the periplasmic trehalase of *Escherichia coli* K12. Mol. Gen. Genet. 217, 347–354. 10.1007/BF024649032671658

[B51] HaganE. C.MobleyH. L. (2009). Haem acquisition is facilitated by a novel receptor Hma and required by uropathogenic *Escherichia coli* for kidney infection. Mol. Microbiol. 71, 79–91. 10.1111/j.1365-2958.2008.06509.x19019144PMC2736550

[B52] HandW. L.SmithJ. W.SanfordJ. P. (1971). The antibacterial effect of normal and infected urinary bladder. J. Lab. Clin. Med. 77, 605–615. 4928903

[B53] HannanT. J.MysorekarI. U.HungC. S.Isaacson-SchmidM. L.HultgrenS. J. (2010). Early severe inflammatory responses to uropathogenic *E. coli* predispose to chronic and recurrent urinary tract infection. PLoS Pathog. 6:e1001042. 10.1371/journal.ppat.100104220811584PMC2930321

[B54] HannanT. J.TotsikaM.MansfieldK. J.MooreK. H.SchembriM. A.HultgrenS. J. (2012). Host-pathogen checkpoints and population bottlenecks in persistent and intracellular uropathogenic *Escherichia coli* bladder infection. FEMS Microbiol. Rev. 36, 616–648. 10.1111/j.1574-6976.2012.00339.x22404313PMC3675774

[B55] HåversenL. A.EngbergI.BaltzerL.DolphinG.HansonL. A.Mattsby-BaltzerI. (2000). Human lactoferrin and peptides derived from a surface-exposed helical region reduce experimental *Escherichia coli* urinary tract infection in mice. Infect. Immun. 68, 5816–5823. 10.1128/IAI.68.10.5816-5823.200010992490PMC101542

[B56] HoodM. I.SkaarE. P. (2012). Nutritional immunity: transition metals at the pathogen-host interface. Nat. Rev. Microbiol. 10, 525–537. 10.1038/nrmicro283622796883PMC3875331

[B57] HootonT. M.ScholesD.StapletonA. E.RobertsP. L.WinterC.GuptaK.. (2000). A prospective study of asymptomatic bacteriuria in sexually active young women. N. Engl. J. Med. 343, 992–997. 10.1056/NEJM20001005343140211018165

[B58] HryckowianA. J.BaisaG. A.SchwartzK. J.WelchR. A. (2015). dsdA does not affect colonization of the murine urinary tract by *Escherichia coli* CFT073. PLoS ONE 10:e0138121 10.1371/journal.pone.013812126366567PMC4569052

[B59] HuangY.NishikawaT.SatohK.IwataT.FukushimaT.SantaT.. (1998). Urinary excretion of D-serine in human: comparison of different ages and species. Biol. Pharm. Bull. 21, 156–162. 10.1248/bpb.21.1569514611

[B60] HullR.RudyD.DonovanW.SvanborgC.WieserI.StewartC.. (2000). Urinary tract infection prophylaxis using *Escherichia coli* 83972 in spinal cord injured patients. J. Urol. 163, 872–877. 10.1016/S0022-5347(05)67823-810687996

[B61] IpeD. S.Ben ZakourN. L.SullivanM. J.BeatsonS. A.UlettK. B.BenjaminW. H.. (2016). Discovery and characterization of human urine utilization by asymptomatic bacteriuria *streptococcus agalactiae*. Infect. Immun. 84, 307–319. 10.1128/IAI.00938-1526553467PMC4694007

[B62] IpeD. S.SundacL.BenjaminW. H.Jr.MooreK. H.UlettG. C. (2013). Asymptomatic bacteriuria: prevalence rates of causal microorganisms, etiology of infection in different patient populations, and recent advances in molecular detection. FEMS Microbiol. Lett. 346, 1–10. 10.1111/1574-6968.1220423808987

[B63] IsaacsonL. C. (1969). Urinary composition in calcific nephrolithiasis. Invest. Urol. 6, 356–363. 5773520

[B64] JainN.KohliR.CookE.GialanellaP.ChangT.FriesB. C. (2007). Biofilm formation by and antifungal susceptibility of Candida isolates from urine. Appl. Environ. Microbiol. 73, 1697–1703. 10.1128/AEM.02439-0617261524PMC1828833

[B65] JärvisaloJ.OlkinuoraM.KiilunenM.KivistöH.RistolaP.TossavainenA.. (1992). Urinary and blood manganese in occupationally nonexposed populations and in manual metal arc welders of mild steel. Int. Arch. Occup. Environ. Health 63, 495–501. 10.1007/BF005721161577529

[B66] JohnsonJ. R.ClabotsC.RosenH. (2006). Effect of inactivation of the global oxidative stress regulator oxyR on the colonization ability of *Escherichia coli* O1:K1:H7 in a mouse model of ascending urinary tract infection. Infect. Immun. 74, 461–468. 10.1128/IAI.74.1.461-468.200616369002PMC1346679

[B67] KingJ. E.Aal OwaifH. A.JiaJ.RobertsI. S. (2015). Phenotypic heterogeneity in expression of the K1 polysaccharide capsule of uropathogenic *Escherichia coli* and downregulation of the capsule genes during growth in urine. Infect. Immun. 83, 2605–2613. 10.1128/IAI.00188-1525870229PMC4468546

[B68] KlemmP.HancockV.SchembriM. A. (2007). Mellowing out: adaptation to commensalism by *Escherichia coli* asymptomatic bacteriuria strain 83972. Infect. Immun. 75, 3688–3695. 10.1128/IAI.01730-0617502385PMC1951988

[B69] KlemmP.RoosV.UlettG. C.SvanborgC.SchembriM. A. (2006). Molecular characterization of the *Escherichia coli* asymptomatic bacteriuria strain 83972: the taming of a pathogen. Infect. Immun. 74, 781–785. 10.1128/IAI.74.1.781-785.200616369040PMC1346676

[B70] KlineK. A.SchwartzD. J.GilbertN. M.HultgrenS. J.LewisA. L. (2012). Immune modulation by group B Streptococcus influences host susceptibility to urinary tract infection by uropathogenic *Escherichia coli*. Infect. Immun. 80, 4186–4194. 10.1128/IAI.00684-1222988014PMC3497425

[B71] KucheriaR.DasguptaP.SacksS. H.KhanM. S.SheerinN. S. (2005). Urinary tract infections: new insights into a common problem. Postgrad. Med. J. 81, 83–86. 10.1136/pgmj.2004.02303615701738PMC1743204

[B72] KuninC. M.HuaT. H.BakaletzL. O. (1995). Effect of salicylate on expression of flagella by *Escherichia coli* and Proteus, Providencia, and Pseudomonas spp. Infect. Immun. 63, 1796–1799. 772988810.1128/iai.63.5.1796-1799.1995PMC173226

[B73] KuninC. M.HuaT. H.GuerrantR. L.BakaletzL. O. (1994). Effect of salicylate, bismuth, osmolytes, and tetracycline resistance on expression of fimbriae by *Escherichia coli*. Infect. Immun. 62, 2178–2186. 791059110.1128/iai.62.6.2178-2186.1994PMC186495

[B74] KuninC. M.HuaT. H.Van Arsdale WhiteL.VillarejoM. (1992). Growth of *Escherichia coli* in human urine: role of salt tolerance and accumulation of glycine betaine. J. Infect. Dis. 166, 1311–1315. 10.1093/infdis/166.6.13111431248

[B75] LaiminsL. A.RhoadsD. B.AltendorfK.EpsteinW. (1978). Identification of the structural proteins of an ATP-driven potassium transport system in *Escherichia coli*. Proc. Natl. Acad. Sci. U.S.A. 75, 3216–3219. 10.1073/pnas.75.7.3216356049PMC392745

[B76] LandeteJ. M.García-HaroL.BlascoA.ManzanaresP.BerbegalC.MonederoV.. (2010). Requirement of the *Lactobacillus casei* MaeKR two-component system for L-malic acid utilization via a malic enzyme pathway. Appl. Environ. Microbiol. 76, 84–95. 10.1128/AEM.02145-0919897756PMC2798650

[B77] La RosaS. L.DiepD. B.NesI. F.BredeD. A. (2012). Construction and application of a luxABCDE reporter system for real-time monitoring of *Enterococcus faecalis* gene expression and growth. Appl. Environ. Microbiol. 78, 7003–7011. 10.1128/AEM.02018-1222843522PMC3457518

[B78] LeeS. C.HutchinsonJ. M.InnK. G.TheinM. (1995). An intercomparison study of 237Np determination in artificial urine samples. Health Phys. 68, 350–358. 10.1097/00004032-199503000-000077860306

[B79] LehmanS. M.DonlanR. M. (2015). Bacteriophage-mediated control of a two-species biofilm formed by microorganisms causing catheter-associated urinary tract infections in an *in vitro* urinary catheter model. Antimicrob. Agents Chemother. 59, 1127–1137. 10.1128/AAC.03786-1425487795PMC4335898

[B80] LeonhardtK. O.LandesR. R. (1963). Oxygen tension of the urine and renal structures. Preliminary report of clinical findings. N. Engl. J. Med. 269, 115–121. 10.1056/NEJM19630718269030113929733

[B81] LombergH.HansonL. A.JacobssonB.JodalU.LefflerH.EdénC. S. (1983). Correlation of P blood group, vesicoureteral reflux, and bacterial attachment in patients with recurrent pyelonephritis. N. Engl. J. Med. 308, 1189–1192. 10.1056/NEJM1983051930820036341837

[B82] LowY. L.JakubovicsN. S.FlatmanJ. C.JenkinsonH. F.SmithA. W. (2003). Manganese-dependent regulation of the endocarditis-associated virulence factor EfaA of *Enterococcus faecalis*. J. Med. Microbiol. 52, 113–119. 10.1099/jmm.0.05039-012543916

[B83] MabbettA. N.UlettG. C.WattsR. E.TreeJ. J.TotsikaM.OngC. L.. (2009). Virulence properties of asymptomatic bacteriuria *Escherichia coli*. Int. J. Med. Microbiol. 299, 53–63. 10.1016/j.ijmm.2008.06.00318706859

[B84] MansouriM. D.DarouicheR. O. (2008). *In-vitro* activity and *in-vivo* efficacy of catheters impregnated with chloroxylenol and thymol against uropathogens. Clin. Microbiol. Infect. 14, 190–192. 10.1111/j.1469-0691.2007.01894.x18042195

[B85] MartinoP. D.FursyR.BretL.SundararajuB.PhillipsR. S. (2003). Indole can act as an extracellular signal to regulate biofilm formation of *Escherichia coli* and other indole-producing bacteria. Can. J. Microbiol. 49, 443–449. 10.1139/w03-05614569285

[B86] MayrovitzH. N.SimsN. (2001). Biophysical effects of water and synthetic urine on skin. Adv. Skin Wound Care 14, 302–308. 10.1097/00129334-200111000-0001311794441

[B87] MeuryJ.RobinA.Monnier-ChampeixP. (1985). Turgor-controlled K+ fluxes and their pathways in *Escherichia coli*. Eur. J. Biochem. 151, 613–619. 10.1111/j.1432-1033.1985.tb09148.x3896791

[B88] MillerJ. D.RandolphA. D.DrachG. W. (1977). Observations upon calcium oxalate crystallization kinetics in simulated urine. J. Urol. 117, 342–345. 1426610.1016/s0022-5347(17)58453-0

[B89] MinuthJ. N.MusherD. M.ThorsteinssonS. B. (1976). Inhibition of the antibacterial activity of gentamicin by urine. J. Infect. Dis. 133, 14–21. 10.1093/infdis/133.1.141450

[B90] NegriM.SilvaS.BredaD.HenriquesM.AzeredoJ.OliveiraR. (2012). Candida tropicalis biofilms: effect on urinary epithelial cells. Microb. Pathog. 53, 95–99. 10.1016/j.micpath.2012.05.00622627049

[B91] NegriM.SilvaS.CapociI. R.AzeredoJ.HenriquesM. (2015). Candida tropicalis biofilms: biomass, metabolic activity and secreted aspartyl proteinase production. Mycopathologia. 10.1007/s11046-015-9964-4. [Epub ahead of print].26572148

[B92] NegriM.SilvaS.HenriquesM.AzeredoJ.SvidzinskiT.OliveiraR. (2011). Candida tropicalis biofilms: artificial urine, urinary catheters and flow model. Medical Mycology 49, 739–747. 10.3109/13693786.2011.56061921366508

[B93] NickelJ. C.RuseskaI.WrightJ. B.CostertonJ. W. (1985). Tobramycin resistance of *Pseudomonas aeruginosa* cells growing as a biofilm on urinary catheter material. Antimicrob. Agents Chemother. 27, 619–624. 10.1128/AAC.27.4.6193923925PMC180108

[B94] NicolleL. E. (1997). Asymptomatic bacteriuria in the elderly. Infect. Dis. Clin. North Am. 11, 647–662. 10.1016/S0891-5520(05)70378-09378928

[B95] NicolleL. E. (1999). Urinary infections in the elderly: symptomatic of asymptomatic? Int. J. Antimicrob. Agents 11, 265–268. 1039498110.1016/s0924-8579(99)00028-x

[B96] NicolleL. E. (2014). Asymptomatic bacteriuria. Curr. Opin. Infect. Dis. 27, 90–96. 10.1097/QCO.000000000000001924275697

[B97] NicolleL. E.BradleyS.ColganR.RiceJ. C.SchaefferA.HootonT. M. (2005). Infectious Diseases Society of America guidelines for the diagnosis and treatment of asymptomatic bacteriuria in adults. Clin. Infect. Dis. 40, 643–654. 10.1086/42750715714408

[B98] NielubowiczG. R.MobleyH. L. (2010). Host-pathogen interactions in urinary tract infection. Nat. Rev. Urol. 7, 430–441. 10.1038/nrurol.2010.10120647992

[B99] O'gradyF.CattellW. R. (1966a). Kinetics of urinary tract infection. I. Upper urinary tract. Br. J. Urol. 38, 149–155. 593476810.1111/j.1464-410x.1966.tb09693.x

[B100] O'gradyF.CattellW. R. (1966b). Kinetics of urinary tract infection. II. The bladder. Br. J. Urol. 38, 156–162. 593476910.1111/j.1464-410x.1966.tb09694.x

[B101] O'gradyF.PenningtonJ. H. (1966). Bacterial growth in an *in vitro* system simulating conditions in the urinary bladder. Br. J. Exp. Pathol. 47, 152–157. 5943816PMC2094579

[B102] OngC. L.BeatsonS. A.McEwanA. G.SchembriM. A. (2009). Conjugative plasmid transfer and adhesion dynamics in an *Escherichia coli* biofilm. Appl. Environ. Microbiol. 75, 6783–6791. 10.1128/AEM.00974-0919717626PMC2772452

[B103] OngC. L.BeatsonS. A.TotsikaM.ForestierC.McEwanA. G.SchembriM. A. (2010). Molecular analysis of type 3 fimbrial genes from *Escherichia coli*, Klebsiella and Citrobacter species. BMC Microbiol. 10:183. 10.1186/1471-2180-10-18320576143PMC2900259

[B104] OpalkoF. J.AdairJ. H.KhanS. R. (1997). Heterogeneous nucleation of calcium oxalate trihydrate in artificial urine by constant composition. J. Cryst. Growth 181, 410–417. 10.1016/S0022-0248(97)00222-4

[B105] PätzoldR.SchieberA.BrücknerH. (2005). Gas chromatographic quantification of free D-amino acids in higher vertebrates. Biomed. Chromatogr. 19, 466–473. 10.1002/bmc.51516037932

[B106] PhuengkhamH.NasongklaN. (2015). Development of antibacterial coating on silicone surface via chlorhexidine-loaded nanospheres. J. Mater. Sci. Mater. Med. 26:78. 10.1007/s10856-015-5418-225631275

[B107] PutnamD. F.Company-WestM. D. A.CenterL. R.AeronauticsU. S. N.AdministrationS. (1971). Composition and Concentrative Properties of Human Urine. Washington, DC: National Aeronautics and Space Administration.

[B108] RaffiH. S.BatesJ. M.Jr.LaszikZ.KumarS. (2005). Tamm-Horsfall protein acts as a general host-defense factor against bacterial cystitis. Am. J. Nephrol. 25, 570–578. 10.1159/00008899016244464

[B109] RagnarsdóttirB.SvanborgC. (2012). Susceptibility to acute pyelonephritis or asymptomatic bacteriuria: host-pathogen interaction in urinary tract infections. Pediatric Nephrol. 27, 2017–2029. 10.1007/s00467-011-2089-122327887

[B110] RaneH. S.BernardoS. M.HowellA. B.LeeS. A. (2014). Cranberry-derived proanthocyanidins prevent formation of Candida albicans biofilms in artificial urine through biofilm- and adherence-specific mechanisms. J. Antimicrob. Chemother. 69, 428–436. 10.1093/jac/dkt39824114570PMC3937597

[B111] RobertsonW. G.PeacockM.NordinB. E. (1968). Activity products in stone-forming and non-stone-forming urine. Clin. Sci. 34, 579–594. 5666884

[B112] RobertsonW. G.ScurrD. S. (1986). Modifiers of calcium oxalate crystallization found in urine. I. Studies with a continuous crystallizer using an artificial urine. J. Urol. 135, 1322–1326. 242371410.1016/s0022-5347(17)46084-8

[B113] RobertsonW. G.ScurrD. S.BridgeC. M. (1981). Factors influencing the crystallization of calcium-oxalate in urine - critique. J. Cryst. Growth 53, 182–194. 10.1016/0022-0248(81)90064-6

[B114] RobinsonA. V.FisherD. R.HadleyR. T. (1984). Technical Evaluation of Draft ANSI Standard N13.30, Performance Criteria for Radioassay. Richland, WA: Pacific Northwest Laboratory.

[B115] RodgersA. L.WandtM. A. (1991). Influence of ageing, pH and various additives on crystal formation in artificial urine. Scanning Microsc. 5, 697–705. discussion: 705–696. 1808707

[B116] RoeschP. L.RedfordP.BatcheletS.MoritzR. L.PellettS.HaugenB. J.. (2003). Uropathogenic *Escherichia coli* use D-serine deaminase to modulate infection of the murine urinary tract. Mol. Microbiol. 49, 54–67. 10.1046/j.1365-2958.2003.03543.x12823810

[B117] RonaldA.LudwigE. (2001). Urinary tract infections in adults with diabetes. Int. J. Antimicrob. Agents 17, 287–292. 10.1016/S0924-8579(00)00356-311295410

[B118] RoosV.NielsenE. M.KlemmP. (2006a). Asymptomatic bacteriuria *Escherichia coli* strains: adhesins, growth and competition. FEMS Microbiol. Lett. 262, 22–30. 10.1111/j.1574-6968.2006.00355.x16907735

[B119] RoosV.UlettG. C.SchembriM. A.KlemmP. (2006b). The asymptomatic bacteriuria *Escherichia coli* strain 83972 outcompetes uropathogenic *E. coli* strains in human urine. Infect. Immun. 74, 615–624. 10.1128/IAI.74.1.615-624.200616369018PMC1346649

[B120] RoseM. B. (1975). Renal stone formation. The inhibitory effect of urine on calcium oxalate precipitation. Invest. Urol. 12, 428–433. 1120635

[B121] RubinR. H.ShapiroE. D.AndrioleV. T.DavisR. J.StammW. E. (1992). Evaluation of new anti-infective drugs for the treatment of urinary tract infection. Infectious Diseases Society of America and the Food and Drug Administration. Clin. Infect. Dis. 15(Suppl. 1), S216–S227. 10.1093/clind/15.supplement_1.s2161477233

[B122] RudickC. N.BillipsB. K.PavlovV. I.YaggieR. E.SchaefferA. J.KlumppD. J. (2010). Host-pathogen interactions mediating pain of urinary tract infection. J. Infect. Dis. 201, 1240–1249. 10.1086/65127520225955PMC2841043

[B123] RussoT. A.JodushS. T.BrownJ. J.JohnsonJ. R. (1996). Identification of two previously unrecognized genes (guaA and argC) important for uropathogenesis. Mol. Microbiol. 22, 217–229. 10.1046/j.1365-2958.1996.00096.x8930907

[B124] RussoT. A.OlsonR.MacdonaldU.BeananJ.DavidsonB. A. (2015). Aerobactin, but not yersiniabactin, salmochelin, or enterobactin, enables the growth/survival of hypervirulent (hypermucoviscous) *Klebsiella pneumoniae ex vivo* and *in vivo*. Infect. Immun. 83, 3325–3333. 10.1128/IAI.00430-1526056379PMC4496593

[B125] RyallR. L.HarnettR. M.HibberdC. M.MazzachiB. C.MazzachiR. D.MarshallV. R. (1987). Urinary risk factors in calcium oxalate stone disease: comparison of men and women. Br. J. Urol. 60, 480–488. 10.1111/j.1464-410X.1987.tb05025.x3427328

[B126] SäemannM. D.WeichhartT.HörlW. H.ZlabingerG. J. (2005). Tamm-Horsfall protein: a multilayered defence molecule against urinary tract infection. Eur. J. Clin. Invest. 35, 227–235. 10.1111/j.1365-2362.2005.01483.x15816991

[B127] SakinçT.MichalskiN.KleineB.GatermannS. G. (2009). The uropathogenic species *Staphylococcus saprophyticus* tolerates a high concentration of D-serine. FEMS Microbiol. Lett. 299, 60–64. 10.1111/j.1574-6968.2009.01731.x19674114

[B128] SakoS.KariyamaR.MitsuhataR.YamamotoM.WadaK.IshiiA.. (2014). Molecular epidemiology and clinical implications of metallo-beta-lactamase-producing *Pseudomonas aeruginosa* isolated from urine. Acta Med. Okayama 68, 89–99. 2474378410.18926/AMO/52405

[B129] SalvadorE.WagenlehnerF.KohlerC. D.MellmannA.HackerJ.SvanborgC.. (2012). Comparison of asymptomatic bacteriuria *Escherichia coli* isolates from healthy individuals versus those from hospital patients shows that long-term bladder colonization selects for attenuated virulence phenotypes. Infect. Immun. 80, 668–678. 10.1128/IAI.06191-1122104113PMC3264318

[B130] SamaranayakeY. H.BandaraH. M.CheungB. P.YauJ. Y.YeungS. K.SamaranayakeL. P. (2014). Enteric Gram-negative bacilli suppress Candida biofilms on Foley urinary catheters. APMIS 122, 47–58. 10.1111/apm.1209823656511

[B131] SaradaB.SatyanarayanaU. (1991). Urinary composition in men and women and the risk of urolithiasis. Clin. Biochem. 24, 487–490. 10.1016/S0009-9120(05)80007-41773489

[B132] SchneebergerC.GeerlingsS. E.MiddletonP.CrowtherC. A. (2012). Interventions for preventing recurrent urinary tract infection during pregnancy. Cochrane Database Syst. Rev. 11:CD009279. 10.1002/14651858.CD009279.pub223152271

[B133] SchneebergerC.KazemierB. M.GeerlingsS. E. (2014). Asymptomatic bacteriuria and urinary tract infections in special patient groups: women with diabetes mellitus and pregnant women. Curr. Opin. Infect. Dis. 27, 108–114. 10.1097/QCO.000000000000002824296584

[B134] ShaykhutdinovR. A.MacinnisG. D.DowlatabadiR.WeljieA. M.VogelH. J. (2009). Quantitative analysis of metabolite concentrations in human urine samples using 13C{1H} NMR spectroscopy. Metabolomics 5, 307–317. 10.1007/s11306-009-0155-5

[B135] SheewinN. S. (2011). Urinary tract infection. Medicine 39, 384–389. 10.1016/j.mpmed.2011.04.00325986163

[B136] ShepardB. D.GilmoreM. S. (2002). Differential expression of virulence-related genes in *Enterococcus faecalis* in response to biological cues in serum and urine. Infect. Immun. 70, 4344–4352. 10.1128/IAI.70.8.4344-4352.200212117944PMC128128

[B137] Shields-CutlerR. R.CrowleyJ. R.HungC. S.StapletonA. E.AldrichC. C.MarschallJ.. (2015). Human urinary composition controls antibacterial activity of siderocalin. J. Biol. Chem. 290, 15949–15960. 10.1074/jbc.M115.64581225861985PMC4481200

[B138] SilvaS.NegriM.HenriquesM.OliveiraR.WilliamsD.AzeredoJ. (2010). Silicone colonization by non-Candida albicans Candida species in the presence of urine. J. Med. Microbiol. 59, 747–754. 10.1099/jmm.0.017517-020299506

[B139] SnyderJ. A.HaugenB. J.BucklesE. L.LockatellC. V.JohnsonD. E.DonnenbergM. S.. (2004). Transcriptome of uropathogenic *Escherichia coli* during urinary tract infection. Infect. Immun. 72, 6373–6381. 10.1128/IAI.72.11.6373-6381.200415501767PMC523057

[B140] SobelJ. D. (1985). New aspects of pathogenesis of lower urinary tract infections. Urology 26, 11–16. 3904135

[B141] Soler-GarcíaA. A.JohnsonD.HathoutY.RayP. E. (2009). Iron-related proteins: candidate urine biomarkers in childhood HIV-associated renal diseases. Clin. J. Am. Soc. Nephrol. 4, 763–771. 10.2215/CJN.020060819279121PMC2666435

[B142] StameyT. A.MiharaG. (1980). Observations on the growth of urethral and vaginal bacteria in sterile urine. J. Urol. 124, 461–463. 742058610.1016/s0022-5347(17)55496-8

[B143] StorerM. K.Hibbard-MellesK.DavisB.ScotterJ. (2011). Detection of volatile compounds produced by microbial growth in urine by selected ion flow tube mass spectrometry (SIFT-MS). J. Microbiol. Methods 87, 111–113. 10.1016/j.mimet.2011.06.01221741416

[B144] StrømA. R.KaasenI. (1993). Trehalose metabolism in *Escherichia coli*: stress protection and stress regulation of gene expression. Mol. Microbiol. 8, 205–210. 10.1111/j.1365-2958.1993.tb01564.x8391102

[B145] StyrvoldO. B.StrømA. R. (1991). Synthesis, accumulation, and excretion of trehalose in osmotically stressed Escherichia coli K-12 strains: influence of amber suppressors and function of the periplasmic trehalase. J. Bacteriol. 173, 1187–1192. 182508210.1128/jb.173.3.1187-1192.1991PMC207241

[B146] SundénF.HåkanssonL.LjunggrenE.WulltB. (2006). Bacterial interference–is deliberate colonization with *Escherichia coli* 83972 an alternative treatment for patients with recurrent urinary tract infection? Int. J. Antimicrob. Agents 28(Suppl. 1), S26–S29. 10.1016/j.ijantimicag.2006.05.00716843646

[B147] SvanborgC.BergstenG.FischerH.GodalyG.GustafssonM.KarpmanD.. (2006). Uropathogenic *Escherichia coli* as a model of host-parasite interaction. Curr. Opin. Microbiol. 9, 33–39. 10.1016/j.mib.2005.12.01216406777

[B148] TanC. K.CareyA. J.CuiX.WebbR. I.IpeD.CrowleyM.. (2012). Genome-wide mapping of cystitis due to *Streptococcus agalactiae* and *Escherichia coli* in mice identifies a unique bladder transcriptome that signifies pathogen-specific antimicrobial defense against urinary tract infection. Infect. Immun. 80, 3145–3160. 10.1128/IAI.00023-1222733575PMC3418756

[B149] TasevskaN.RunswickS. A.McTaggartA.BinghamS. A. (2005). Urinary sucrose and fructose as biomarkers for sugar consumption. Cancer Epidemiol. Biomarkers Prevent. 14, 1287–1294. 10.1158/1055-9965.EPI-04-082715894688

[B150] TielenP.RosinN.MeyerA. K.DohntK.HaddadI.JänschL.. (2013). Regulatory and metabolic networks for the adaptation of *Pseudomonas aeruginosa* biofilms to urinary tract-like conditions. PLoS ONE 8:e71845. 10.1371/journal.pone.007184523967252PMC3742457

[B151] TorffvitO.AgardhC. D. (1993). Tubular secretion of Tamm-Horsfall protein is decreased in type 1 (insulin-dependent) diabetic patients with diabetic nephropathy. Nephron 65, 227–231. 10.1159/0001874798247185

[B152] TorzewskaA.BudzynskaA.Bialczak-KokotM.RózalskiA. (2014). *In vitro* studies of epithelium-associated crystallization caused by uropathogens during urinary calculi development. Microb. Pathog. 71–72, 25–31. 10.1016/j.micpath.2014.04.00724803200

[B153] TorzewskaA.RózalskiA. (2014). *In vitro* studies on the role of glycosaminoglycans in crystallization intensity during infectious urinary stones formation. APMIS 122, 505–511. 10.1111/apm.1219124164670

[B154] TorzewskaA.RózalskiA. (2015). Various intensity of Proteus mirabilis-induced crystallization resulting from the changes in the mineral composition of urine. Acta Biochim. Pol. 62, 127–132. 10.18388/abp.2014_88225654361

[B155] TorzewskaA.StaczekP.RózalskiA. (2003). Crystallization of urine mineral components may depend on the chemical nature of Proteus endotoxin polysaccharides. J. Med. Microbiol. 52, 471–477. 10.1099/jmm.0.05161-012748265

[B156] UlettG. C.TotsikaM.SchaaleK.CareyA. J.SweetM. J.SchembriM. A. (2013). Uropathogenic *Escherichia coli* virulence and innate immune responses during urinary tract infection. Curr. Opin. Microbiol. 16, 100–107. 10.1016/j.mib.2013.01.00523403118

[B157] UppuluriP.DinakaranH.ThomasD. P.ChaturvediA. K.Lopez-RibotJ. L. (2009). Characteristics of *Candida albicans* biofilms grown in a synthetic urine medium. J. Clin. Microbiol. 47, 4078–4083. 10.1128/JCM.01377-0919794044PMC2786631

[B158] VebøH. C.SolheimM.SnipenL.NesI. F.BredeD. A. (2010). Comparative genomic analysis of pathogenic and probiotic *Enterococcus faecalis* isolates, and their transcriptional responses to growth in human urine. PLoS ONE 5:e12489. 10.1371/journal.pone.001248920824220PMC2930860

[B159] VejborgR. M.de EvgrafovM. R.PhanM. D.TotsikaM.SchembriM. A.HancockV. (2012). Identification of genes important for growth of asymptomatic bacteriuria *Escherichia coli* in urine. Infect. Immun. 80, 3179–3188. 10.1128/IAI.00473-1222753377PMC3418751

[B160] WattsR. E.HancockV.OngC. L.VejborgR. M.MabbettA. N.TotsikaM.. (2010). *Escherichia coli* isolates causing asymptomatic bacteriuria in catheterized and noncatheterized individuals possess similar virulence properties. J. Clin. Microbiol. 48, 2449–2458. 10.1128/JCM.01611-0920444967PMC2897502

[B161] WattsR. E.TanC. K.UlettG. C.CareyA. J.TotsikaM.IdrisA.. (2012a). *Escherichia coli* 83972 expressing a P fimbriae oligosaccharide receptor mimic impairs adhesion of uropathogenic *E. coli*. J. Infect. Dis. 206, 1242–1249. 10.1093/infdis/jis49322872729

[B162] WattsR. E.TotsikaM.ChallinorV. L.MabbettA. N.UlettG. C.De VossJ. J.. (2012b). Contribution of siderophore systems to growth and urinary tract colonization of asymptomatic bacteriuria *Escherichia coli*. Infect. Immun. 80, 333–344. 10.1128/IAI.05594-1121930757PMC3255690

[B163] WeinbergE. D. (1978). Iron and infection. Microbiol. Rev. 42, 45–66. 37957210.1128/mr.42.1.45-66.1978PMC281418

[B164] Wenzler-RötteleS.DettenkoferM.Schmidt-EisenlohrE.GregersenA.Schulte-MontingJ.TvedeM. (2006). Comparison in a laboratory model between the performance of a urinary closed system bag with double non-return valve and that of a single valve system. Infection 34, 214–218. 10.1007/s15010-006-5626-216896580

[B165] WernliL.BonkatG.GasserT. C.BachmannA.BraissantO. (2013). Use of isothermal microcalorimetry to quantify the influence of glucose and antifungals on the growth of *Candida albicans* in urine. J. Appl. Microbiol. 115, 1186–1193. 10.1111/jam.1230623865534

[B166] WilksS. A.FaderM. J.KeevilC. W. (2015). Novel insights into the *Proteus mirabilis* crystalline biofilm using real-time imaging. PLoS ONE 10:e0141711. 10.1371/journal.pone.014171126516766PMC4627822

[B167] WishartD. S.KnoxC.GuoA. C.EisnerR.YoungN.GautamB.. (2009). HMDB: a knowledgebase for the human metabolome. Nucleic Acids Res. 37, D603–D610. 10.1093/nar/gkn81018953024PMC2686599

[B168] WulltB. (2003). The role of P fimbriae for *Escherichia coli* establishment and mucosal inflammation in the human urinary tract. Int. J. Antimicrob. Agents 21, 605–621. 10.1016/S0924-8579(02)00328-X13678032

[B169] WulltB.ConnellH.RöllanoP.MånssonW.ColleenS.SvanborgC. (1998). Urodynamic factors influence the duration of *Escherichia coli* bacteriuria in deliberately colonized cases. J. Urol. 159, 2057–2062. 10.1016/S0022-5347(01)63246-49598517

[B170] ZdziarskiJ.BrzuszkiewiczE.WulltB.LiesegangH.BiranD.VoigtB.. (2010). Host imprints on bacterial genomes–rapid, divergent evolution in individual patients. PLoS Pathog. 6:e1001078. 10.1371/journal.ppat.100107820865122PMC2928814

